# Effect Evaluation of Cardiac Resynchronization Therapy in Elderly Patients with Heart Failure by Ultrasound Image under QuickOpt Algorithm

**DOI:** 10.1155/2022/8680446

**Published:** 2022-06-07

**Authors:** Na Hu, Na Yi, Huiqiong Yang

**Affiliations:** ^1^Department of Cardiovascular Medicine, Changsha Fourth Hospital, Changsha, 410000 Hunan, China; ^2^General Medicine, Changsha Fourth Hospital, Changsha, 410000 Hunan, China

## Abstract

This research was aimed at analyzing the application value of echocardiography and QuickOpt algorithm in optimizing parameters of cardiac resynchronization therapy (CRT) in elderly patients with heart failure. 50 elderly patients who were diagnosed with chronic heart failure and underwent CRT were chosen as the research objects. According to the different optimization methods, the patients were divided into the echocardiography group and QuickOpt algorithm group, 25 cases in each group. The general data, optimized intervals, corresponding maximum aortic velocity time integrals (aVTIs), cardiac ultrasound indicators, and ventricular arrhythmia episodes of the patients in the two groups were analyzed. The results showed that there was no significant difference in the optimized sensed atrioventricular (SAV), paced atrioventricular (PAV), and ventricle to ventricle (VV) intervals and the corresponding aVTIs obtained by echocardiography and QuickOpt (*P* > 0.05). The consistency analysis revealed that the aVTIs in the SAV, PAV, and VV intervals presented a good consistency (*P* < 0.01), which were obtained by the echocardiography and QuickOpt functional optimization; the concordance correlation coefficient (CCC) in them was 96.16%, 98.03%, and 95.48%, respectively. The left ventricular ejection fraction (LVEF) showed an increasing trend over time in both groups, while the left ventricular end systolic volume (LVESV), left ventricular end diastolic volume (LVEDV), and morphological right ventricle (MRV) showed the downward trends over time, and the differences between two groups were not significant (*P* > 0.05). For the premature ventricular contraction (PVC) of ventricular arrhythmia episodes, there was no significant difference between the two groups in *log* (PVCs) and *log* (PVC runs) (*P* > 0.05). It was also found that both echocardiography and QuickOpt algorithm could improve the cardiac function of patients with heart failure significantly and reduce ventricular arrhythmia episodes and ventricular remodeling via optimized CRT; there was no difference in the improvement effect of the two optimization methods. However, echocardiography was inferior to QuickOpt algorithm in terms of time-consuming optimization in the intervals. This provided a reference for the clinical diagnosis and treatment of elderly patients with heart failure.

## 1. Introduction

Heart failure refers to the syndrome dominated by circulatory dysfunction, which caused by that the myocardial diastolic and/or systolic dysfunction and insufficient cardiac output cannot maintain tissue metabolism with moderate venous return [1–3]. In clinical practice, heart failure is characterized by decreased cardiac output, decreased tissue blood perfusion, and pulmonary circulatory congestion and/or systemic venous congestion, so it is also called congestive heart failure or cardiac insufficiency [4, 5]. The main clinical manifestations of patients with heart failure are dyspnea, restricted physical activity, fluid retention, and so on. Depending on the locations of the heart failure, the clinical manifestations may be different in patients with left heart failure and right heart failure [6], but it is mainly manifested as a syndrome caused by pulmonary circulatory congestion and decreased cardiac output. The symptoms of left heart failure include exertional dyspnea, orthopnea, paroxysmal dyspnea at night, coughing with pink foamy sputum, hemoptysis, and other more acute pulmonary edema manifestations [7–9]. Right heart failure is the syndrome mainly in which the obstruction of systemic venous return causes congestion and hypoxia in various organs, and the major clinical manifestations are anorexia, nausea, and vomiting caused by long-term gastrointestinal congestion. Cardiac resynchronization therapy (CRT), also known as biventricular pacing, is to increase left ventricular pacing on the basis of traditional pacing. Through CRT, the patients with heart failure could be treated whose ventricular contractions are not synchronized [10, 11]. As CRT can improve patients' cardiac function, exercise tolerance, and quality of life, it is a milestone breakthrough in the history of heart failure treatment.

Clinically, physical examinations are generally used to find signs of heart failure in patients. In addition, there are troponin, electrocardiogram, echocardiography, X-ray examination, cardiac magnetic resonance, cardiopulmonary exercise test, etc., [12–14] can be applied for the diagnosis. If necessary, invasive examinations such as coronary angiography can also be considered to confirm the diagnosis. Echocardiography can accurately evaluate the size changes of the heart chambers and the structure and function of cardiac valves, to assess the cardiac function and determine the cause easily and quickly, so it becomes the most important instrumental examination for the diagnosis of heart failure [15]. However, the device needs to be put into the human body; it will make the patients feel uncomfortable and even cause complications. Therefore, patients with ulcers in the esophagus and stomach or severe arrhythmia are not suitable for echocardiography. The QuickOpt is a method to optimize the parameters of CRT using intracavitary electrocardiogram. It overcomes the above shortcomings to a certain extent, and it saves follow-up time and technical cost for its simple operation. Thus, it is expected to be a routine method for postoperative optimization clinically for specific patients [16]. Therefore, 50 elderly patients with chronic heart failure concurrently treated with CRT were the research samples. These samples were divided into echocardiography group (25 cases) and QuickOpt algorithm group (25 cases). It was to further explore the evaluation performances of echocardiography and the traditional method QuickOpt algorithm on the effect of CRT in elderly patients with heart failure.

## 2. Materials and Methods

### 2.1. Research Objects

Fifty elderly patients who were diagnosed with chronic heart failure and underwent CRT in hospital from October 2019 to February 2021 were chosen as the research objects. With different optimization methods, they were divided into the echocardiography group and QuickOpt algorithm group of 25 patients in each. This study had been approved by ethics committee of hospital, and the patients and their families signed the informed consents.

The included patients must suffer from the refractory congestive heart failure, and the left ventricular end-diastolic inner diameter was greater than or equal to 55 mm. The surface electrocardiogram result was greater than 120 ms under QRS wave complex, and the left ventricular ejection fraction (LVEF) was less than 35%. What is more, they got a successful CRT. Patients with persistent atrial fibrillation, an autonomous heart rate of less than 40 f/min^−1^, complete atrioventricular block, mental illness, or allergic constitution were excluded.

### 2.2. Echocardiography Optimization

Digital color Doppler ultrasound diagnostic apparatus with 3.5 mHz probe was applied in this study. The left ventricular end systolic volume (LVESV), left ventricular end diastolic volume (LVEDV), and morphological right ventricle (MRV) were measured through Simpson method, and the LVEF was also calculated.

Data collection was done by the same physician, and the optimizations of sensed atrioventricular (SAV), paced atrioventricular (PAV), and ventricle to ventricle (VV) intervals were carried out. For the SAV interval optimization, the pacing heart rate was set to be less than the autonomous heart rate; then, when the SAV interval was 160, 140, 120, 100, 80, and 60 ms, respectively, the optimized SAV intervals and the maximum aortic blood flow velocity integrals (aVTIs) were obtained. For the PAV interval optimization, the pacing heart rate was set as about 5-10 f/min^−1^, which was greater than the autonomous heart rate. As the PAV interval was 210, 190, 170, 150, 130, and 110 ms, respectively, the optimized PAV intervals and the corresponding aVTIs were worked out. For the VV interval optimization, the pacing heart rate was set less than the autonomous heart rate, and the VV interval was set as 70, 50, 30, and 10 ms, respectively, in the left ventricle and 10, 30, 50, and 70 ms, respectively, in the right ventricle. With the optimized SAV intervals obtained, the optimized VV intervals and its corresponding aVTIs were worked out.

### 2.3. QuickOpt Algorithm Optimization

In the programmed state, the QuickOpt [17] was used to obtain the patients' optimized SAV, PAV, and VV intervals. The pacing heart rate was set less than the autonomous heart rate, to obtain the aVTIs for each interval.

### 2.4. Data Collection

The general preoperative information of patients was collected, including the age, gender, underlying diseases of heart failure, hypertension and other concomitant diseases, blood creatinine, and drug treatment plan. The cardiac function classification of New York Heart Association, QRS duration, and echocardiogram indicators were recorded before and after surgery. In the follow-ups, the patients were readmitted to hospital for heart failure or all-cause deaths and medication regimens were also recorded.

### 2.5. Postoperative Follow-Ups

During the postoperative outpatient follow-ups, the ventricular arrhythmia data saved by the pulse generator was recorded at each follow-up, including the number of premature ventricular contractions (PVCs) and premature ventricular contraction runs (PVC runs). PVC is defined as any ventricular sensing episodes in the refractory and nonrefractory period, which were not accompanied by atrial episodes of pacing, refractory sensing, and nonrefractory sensing before ventricular episodes of pacing, refractory sensing, and nonrefractory sensing. PVC runs are defined as two or more consecutive PVCs that are not accompanied by atrial episodes. The total numbers of PVCs and PVC runs were accumulated, respectively, and divided by the number of follow-up days to obtain the average numbers per day, which was regarded as the number of middle ventricular arrhythmia episodes within six months after the surgery.

### 2.6. Statistical Methods

The data processing was performed by SPSS19.0 in this study. The measurement data was expressed by the mean ± standard deviation ($\bar{x}\pm s$), and the enumeration data was expressed by the percentage (%). The results were tested by the concordance correlation coefficient (CCC). One-way analysis of variance was used for pairwise comparison. Two-sided test was carried out, and the difference was statistically significant at *P* < 0.05.

## 3. Results

### 3.1. General Conditions of All the Patients

As shown in Figure 1 below, among the included patients, 39 were males and 11 were females. 38 cases were ≥65 years old, while 12 cases were <65 years old. 14 cases were caused by ischemic cardiomyopathy, and 36 cases went without that.

### 3.2. General Data Comparison between the Echocardiography and QuickOpt Algorithm Groups

As shown in Figure 2, the general data, postoperative medications, and ultrasound indicators of the patients in both groups were compared, and there was no statistically significant difference (*P* > 0.05). The compared general data included the age, male proportion, and history of diabetes; the postoperative medications included diuretics, digoxin, angiotensin-converting enzyme inhibitors (ACEI)/angiotensin II receptor blockers (ARB), and *β*-receptor blockers; the ultrasound indicators were LVEF, LVESV, LVEDV, and QRS duration (QRSd).

### 3.3. Imaging Data of Patients

Figure 3 shows the echocardiograms of a male case, who was 65 years old. He had oppression in the chest and edemas in both lower extremities while moving after being cold. He had high blood pressure, hyperlipidemia, and burning sensation in the extremities, and the ventricular rate was about 160 f/min^−1^. From the echocardiograms, the LVEF was 50%, the left ventricular end-diastolic inner diameter was 6.6 cm, and there was no obvious valve abnormality.

Figure 4 shows the echocardiograms of a 63-year-old female case, who had a history of stroke, and new atrial fibrillation occurred when she visited the doctors. The echocardiograms revealed decreased left ventricular diastolic function, moderate left ventricular hypertrophy, and mild pulmonary arterial hypertension. In addition, the patient suffered from severe symptoms of fatigue after moving and edemas in both lower extremities.

### 3.4. Comparison of Optimized Intervals and Corresponding aVTIs between Two Groups

In Figure 5(a), the differences in optimized SAV, PAV, and VV intervals between the echocardiography and QuickOpt algorithm groups were not statistically significant (*P* > 0.05).

In Figure 5(b), there was also no statistically significant difference in aVTIs of SAV, PAV, and VV intervals, respectively, between the echocardiography group and QuickOpt algorithm group (*P* > 0.05). The consistency analysis showed that the aVTIs of the SAV, PAV, and VV intervals obtained by the echocardiographic optimization and the QuickOpt functional optimization had good consistency (*P* < 0.01), and the CCC was 96.16%, 98.03%, and 95.48%, respectively.

As shown in Figure 6, the time required for interval optimization by echocardiography was significantly lower than that by QuickOpt algorithm, with the difference statistically significant (*P* < 0.05).

### 3.5. Comparison of Postoperative Clinical Indicators between Two Groups

It is shown in Figure 7 that the LVEF of patients in both the echocardiography group and the QuickOpt algorithm group had an increasing trend over time, 1, 3, and 6 months, respectively, after surgery, but the differences between the two groups were not statistically significant (*P* > 0.05). The LVESV, LVEDV, and MRV of patients in the echocardiography group and the QuickOpt algorithm group 1, 3, and 6 months after surgery showed a downward trend over time, but still, there was not a statistically significant difference between two groups (*P* > 0.05).

In Figure 8, the QRSd of both the echocardiogram group and the QuickOpt algorithm group changed slowly over time, in the 1, 3, and 6 months after surgery, respectively; there was no obvious decrease and no statistically significant difference between the groups (*P* > 0.05).

### 3.6. Comparison of Ventricular Arrhythmia Indicators between the Two Groups

Figure 9 shows the comparison of ventricular arrhythmia indicators in patients in the echocardiography group and QuickOpt algorithm group. It could be observed that the differences of *log* (PVCs) and *log* (PVC runs) of patients' ventricular arrhythmia episodes between the two groups were not statistically significant (*P* > 0.05).

## 4. Discussion

Heart failure is the most important cause of death from cardiovascular diseases. It is not an independent disease, but a common end for multiple cardiac diseases. In clinical practice, CRT is used to treat heart failures generally, as it can improve the life quality and rehabilitation of patients to a certain extent; however, there are still 30% of patients are treated ineffectively. It is generally believed that the main reasons for the poor treatment effect include the evaluation of left ventricular contraction asynchrony, the poor position of the left ventricular electrodes, and the failure of pacing parameter optimization after surgery [18, 19]. Both surface echocardiography and QuickOpt algorithm are methods for CRT parameter optimization, and their influences on the CRT efficacy are unclear so far [20]. In this study, 50 elderly patients with chronic heart failure and treated with CRT were included as the research objects. For the different optimization methods, the patients were divided into the echocardiography group and the QuickOpt algorithm group, with 25 cases, respectively. The general data of patients in the two groups were analyzed, from which the age, male proportion history of diabetes, postoperative medications (diuretics, digoxin, ACEI/ARB, and ꞵ-receptor blockers), and ultrasound indicators (LVEF, LVESV, LVEDV, and QRSd) of patients showed no statistically significant difference between the two groups (*P* > 0.05). Such consistencies of general information provided the feasibility for follow-up research. Besides, the echocardiographic data of some cases were shown in this study, and it could be observed that echocardiography showed the changes in ventricular functions of patients with heart failure clearly, pointing out the patients' condition of heart failure and providing help for the evaluation of clinical treatment [21].

The optimized indicators by echocardiography and QuickOpt algorithm were compared. It was found that the differences of the pairwise optimized SAV, PAV, and VV intervals of two groups were not statistically significant (*P* > 0.05), which suggested the optimized intervals obtained by the echocardiography differed little from those by the QuickOpt algorithm (*P* > 0.05), and both the two methods achieved great optimization effects. There was also no statistically significant difference in aVTIs of the SAV, PAV, and VV intervals between the two groups (*P* > 0.05). It was found via the consistency analysis that the aVTIs of SAV, PAV, and VV intervals obtained by the echocardiography and QuickOpt algorithm had a good consistency (*P* < 0.01), and the CCC was counted as 96.16%, 98.03%, and 95.48%, respectively. Such results were similar to those turned out of Tavazzi et al. [22], indicating that the hemodynamic effects obtained by echocardiographic optimization and QuickOpt parameter optimization were consistent, so both the methods were feasible. The time required for interval optimization by echocardiography was significantly shorter than that by QuickOpt algorithm, going with the statistically significant differences (*P* < 0.05). This was similar to the study results of Mozzini et al. [23]. With the continuous development of myocardial remodeling or reverse remodeling, the optimization of the intervals after CRT implantation is a work needs to be carried out frequently rather than once for all. The quick automatic interval optimization of the QuickOpt algorithm can greatly save time and technical cost due to its simple operations, and it is worthy of clinical application. However, echocardiography has the disadvantages of long time-consuming and poor repeatability [24].

For patients in the echocardiogram group and the QuickOpt algorithm group, the LVEFs 1, 3, and 6 months after surgery showed an upward trend over time, while the LVESV, LVEDV, and MRV showed a decreasing trend, without statistically significant difference between the groups (*P* > 0.05). It was indicated that both echocardiography and QuickOpt algorithm optimization on CRT improved the cardiac function of patients with heart failure greatly, and there was no significant difference in the improvement effect between the two groups [25]. The ventricular arrhythmia episodes after CRT surgery were further analyzed. It could be observed that the differences in *log* (PVCs) and *log* (PVC runs) of ventricular arrhythmia episodes were not statistically significant (*P* > 0.05) between the echocardiography group and the QuickOpt algorithm group. Previous studies showed that the cardiac mechanical remodeling was related to ventricular arrhythmia episodes, as carvedilol was proved to reduce the onset of ventricular arrhythmia episodes while affecting ventricular remodeling in drug trials [26]. This also showed that the optimized CRT by echocardiography and QuickOpt algorithm had no difference in the effects of postoperative ventricular arrhythmia episodes and ventricular remodeling.

## 5. Conclusion

As 50 elderly patients with chronic heart failure and CRT were examined by echocardiography, the optimal interval and corresponding aVTI, echocardiographic indicators, and adverse events were determined. It was suggested from the results that both echocardiography and QuickOpt algorithm had good effects in improving cardiac function and reducing ventricular remodeling in patients with heart failure. But QuickOpt algorithm was superior to echocardiography in time-consuming of the interval optimization. Although the changes of postoperative hemodynamic parameters in patients were explored in this research, there was no long-term follow-up result after the optimization. In the future, a larger amount of patient data would be collected again for a double-blind, multicenter, randomized, and controlled test, and frequent interval optimization would be performed after CRT surgery in patients, so as to analyze whether the two optimization methods have a different effect on the long-term prognosis of patients. All in all, the results of this study gave a reference for the effect evaluation of CRT postoperative parameter optimization in patients with heart failure clinically.

## Figures and Tables

**Figure 1:** Age, gender, and disease causes of patients. (a–c) The genders, ages, and disease causes of patients, respectively.

**Figure 2:** General data comparison between two groups. (a) The comparison of age, male proportion, and history of diabetes; (b) postoperative medications; (c) ultrasound indicators.

**Figure 3:** Echocardiograms of a patient with heart failure. Male, 65 years old.

**Figure 4:** Echocardiograms of a patient with heart failure. Female, 63 years old.

**Figure 5:** Comparisons of optimized intervals and the corresponding aVTIs by echocardiography and QuickOpt algorithm. (a) The comparison of optimized SAV, PAV, and VV intervals; (b) the comparison of aVTIs of SAV, PAV, and VV intervals.

**Figure 6:** Comparison of the time required for interval optimization between two groups. ∗ indicated that the difference compared to the time of the echocardiography group was statistically significant (*P* < 0.05).

**Figure 7:** Comparison of postoperative clinical echocardiographic indicators between two groups. (a–d) The comparisons of LVEF, LVESV, LVEDV, and MRV, respectively.

**Figure 8:** Comparison of postoperative QRSd between the echocardiography group and QuickOpt algorithm group.

**Figure 9:** Comparison of ventricular arrhythmia indicators between the echocardiography group and QuickOpt algorithm group.

## Data Availability

The data used to support the findings of this study are available from the corresponding author upon request.
